The article "ATG4A promotes tumor metastasis by inducing the epithelial-mesenchymal transition and stem-like properties in gastric cells" was retracted in 2025. Reasons: contaminated cell lines or tissues; duplicated images; unreliable data; unreliable results or conclusions.

# ATG4A promotes tumor metastasis by inducing the epithelial-mesenchymal transition and stem-like properties in gastric cells

**DOI:** 10.18632/oncotarget.9827

**Published:** 2016-06-04

**Authors:** Shi-Wei Yang, Yi-Fang Ping, Yu-Xing Jiang, Xiao Luo, Xia Zhang, Xiu-Wu Bian, Pei-Wu Yu

**Affiliations:** ^1^ Department of General Surgery and Center of Minimal Invasive Gastrointestinal Surgery, Southwest Hospital, Third Military Medical University, Chongqing, China; ^2^ Key Laboratory of Tumor Immunopathology of Ministry of Education of China, Third Military Medical University, Chongqing, China; ^3^ Institute of Pathology and Southwest Cancer Center, Southwest Hospital, Third Military Medical University, Chongqing, China

**Keywords:** ATG4A, epithelial-mesenchymal transition, gastric cancer, metastasis, tumor stem cell, Pathology Section

## Abstract

The metastasis of tumor cells to distant organs is an ominous feature of gastric cancer. However, the molecular mechanisms underlying the invasion and metastasis of gastric cancer cells remain elusive. In this study, we found that the expression of ATG4A, an autophagy-regulating molecule, was significantly increased in gastric cancer tissues and was significantlycorrelated with the gastric cancer differentiation degree, tumor invasion and lymph node metastasis. ATG4A over-expression significantly promoted gastric cancer cell migration and invasion *in vitro* and metastasis *in vivo*, as well as promoted gastric cancer cell stem-like properties and the epithelial-mesenchymal transition (EMT) phenotype. By contrast, ATG4A knockdown inhibited the migration, invasion and metastasis of cancer cells, as well as the stem-like properties and EMT phenotype. Mechanistically, ATG4A promotes gastric cancer cell stem-like properties and the EMT phenotype through the activation of Notch signaling not via autophagy, and using the Notch signaling inhibitor DAPT attenuated the effects of ATG4A on gastric cancer cells. Taken together, these findings demonstrated that ATG4A promotes the metastasis of gastric cancer cells via the Notch signaling pathway, which is an autophagy-independent mechanism.

## INTRODUCTION

Gastric cancer is one of the most common malignancies worldwide. There were more than 700,000 deaths due to gastric cancer in 2014, making this disease the third most common cause of cancer death globally [1, 2]. Despite the development and identification of novel anticancer agents and treatment methods over the past decades, almost 50% of gastric cancer patients eventually develop recurrent disease and distant metastasis after surgical treatment [3]. The distant metastasis of gastric cancers is the main cause of more than 90% of patient deaths [4]. Metastasis is a complicated biological cascade that starts with local invasion by tumor cells and continues with migration to distant tissues and organs. Hence, the identification of molecules associated with gastric cancer invasion and metastasis would contribute to the understanding of the mechanisms involved in gastric cancer malignancy, leading to the development of novel biomarkers and therapeutic targets for gastric cancer.

The article "ATG4A promotes tumor metastasis by inducing the epithelial-mesenchymal transition and stem-like properties in gastric cells" was retracted in 2025. Reasons: contaminated cell lines or tissues; duplicated images; unreliable data; unreliable results or conclusions.

Cancer stem cells (CSCs) are a subpopulation of cancer cells that have tumor-initiating capacity [5]. These cells resist apoptosis and DNA damage caused by drugs, which facilitates metastasis [6]. The epithelial-to-mesenchymal transition (EMT) is a crucial program for the invasiveness and metastasis of cancer cells and is typified by the dissolution of cell-cell junctions and the development of individual motile mesenchymal cells with increased mobility. Both decreased levels of E-cadherin and increased levels of N-cadherin are well-established hallmarks of EMT [7]. Empirical evidence concerning the connection of EMT to the emergence of CSCs has been reported recently. Differentiated mammary epithelial cells can undergo EMT to produce CD44^high^ CD24^low^ cells that are similar to breast CSCs [8]. EMT induced by CD8^+^ T cells also results in the formation of CD44^high^ CD24^low^ stem cell-like cells [9]. In addition, stem cells isolated from normal breast tissue or breast cancers express several EMT markers [10]. Therefore, both EMT and stemness are extremely important characteristics for cancer cells to acquire more invasive and metastatic potential. Recent studies have demonstrated that various molecules can trigger EMT and stemness. For instance, miR-22 was proven to be a crucial molecular effector in the promotion EMT and stemness that leads to breast cancer metastasis [11]. Moreover, FBXW7 has been shown to suppress EMT, stemness and metastasis by the mTOR signaling pathway in cholangiocarcinoma cells [12]. However, the molecular mechanism regulating EMT, stemness and metastasis in gastric cancer remains elusive.

Accumulating evidence has suggested that autophagy-regulating molecules are involved in tumorigenesis [13]. ATG4A, a member of the cysteine protease family, plays an important role as an autophagin [14]. The increased expression of ATG4A was observed at the polychromatic erythroid stage, in which autophagy was activated, in differentiating human erythroblasts [15]. Recently, ATG4A overexpression was found in mammospheres, suggesting its potential role in breast cancer stem cell maintenance [16]. In small cell lung cancer, ATG4A was shown to participate in etoposide (VP16) and cisplatin (DDP) resistance [17]. However, the function of ATG4A in gastric cancer remains unclear.

The article "ATG4A promotes tumor metastasis by inducing the epithelial-mesenchymal transition and stem-like properties in gastric cells" was retracted in 2025. Reasons: contaminated cell lines or tissues; duplicated images; unreliable data; unreliable results or conclusions.

In this study, we detected the levels of ATG4A in gastric cancer specimens from 110 patients and compared them with the levels in normal gastric mucosa. Our findings indicate that the expression of ATG4A is significantly higher in gastric cancer tissues and metastatic lymph nodes. Furthermore, we revealed that ATG4A promoted EMT and stemness to induce metastasis in gastric cancer cells through upregulating the Notch signaling pathway.

## RESULTS

### ATG4A predicts the lymph node metastasis of gastric cancer patients

We first evaluated ATG4A expression in gastric cancer specimens from 110 patients and found that ATG4A was predominantly located in the nucleus with a diffuse distribution in the cytoplasm in gastric cancer cells. By contrast, low or undetectable expression of ATG4A was observed in matched non-cancerous tissues (Supplementary Figure S1). The metastatic lymph node showed more intense staining for ATG4A compared to the central tumor areas. Interestingly, the cells in tumor invasion front exhibited significantly higher ATG4A expression than the cells in the central tumor areas (Figure 1A and 1B). Taken together, the results indicated that ATG4A expression is increased in gastric cancer, especially in the tumor invasion front and in lymph node metastatic lesions [18].

The correlation between ATG4A expression and clinicopathological features was further analyzed. As shown in Table 1, the gastric cancer differentiation degree, lymphatic invasion and tumor invasion were significantly associated with ATG4A expression (*P* < 0.05). No significant correlation was observed between ATG4A expression and sex, age and distant metastasis status (*P* > 0.05). Taken together, these results suggest that high expression of ATG4A is associated with more aggressive biological behavior.

**Table 1:** Correlations between ATG4A expression and clinical characteristics of patients with gastric cancer

Clinical factor	ATG4A expression		*P* value
	Low expression (n=35)	High expression (n=75)	
Sex			
Male	17	50	0.070
Female	18	25	
Age(y)			
<60	19	44	0.665
≥60	16	31	
Differentiated degree			
Poor differentiated	9	42	<0.01*
Well +moderate differentiated	26	33	
Lymphoid nodal(N) status			
Absent	19	24	0.025*
Present	16	51	
Tumor (T) invasion			
T1 + T2	21	27	0.018*
T3 + T4	14	48	
Distant metastasis(M) status			
M0	31	70	0.957
M1	4	5	

**Figure 1:** ATG4A is overexpressed in the invasion front and lymph node metastatic lesions of gastric cancers **A.** HE staining and immunohistochemical staining of ATG4A in the tumor center, the invasion front and lymph node metastatic lesions of poor differentiated gastric cancers. **B.** HE staining and immunohistochemical staining of ATG4A in the tumor center, the invasion front and lymph node metastatic lesions of well differentiated gastric cancers. The right bar graph represents scores of ATG4A expression.

The article "ATG4A promotes tumor metastasis by inducing the epithelial-mesenchymal transition and stem-like properties in gastric cells" was retracted in 2025. Reasons: contaminated cell lines or tissues; duplicated images; unreliable data; unreliable results or conclusions.

### ATG4A promotes the migration and invasion of gastric cancer cells *in vitro*

We next investigated the effect of ATG4A on the invasive capacity of gastric cancer cells. The expression of ATG4A in five gastric cancer cell lines was detected. Comparison of various gastric cancer cell lines revealed that MGC-803 cells expressed higher level of ATG4A, SGC-7901 and MKN-47 showed lower ATG4A expression (Figure 2A). SGC-7901 was chose to construct cells stably expressing ATG4A (ATG4A-OE) (Supplementary Figure S2A). In the wound-healing assay, ATG4A-OE cells showed a more invasive phenotype and migrated faster into the wound area than control cells (Figure 2B). Consistently, the number of ATG4A-OE cells migrating into the lower chamber in the transwell chamber invasion assay was higher than that of control cells (Figure 2C). We next knocked down ATG4A expression in MGC-803 cells using shRNA (Supplementary Figure S2B). As expected, MGC-803 cells with ATG4A shRNAs exhibited lower migratory and invasive capacity compared to control cells (Figure 2D and 2E). We further investigate whether ATG4A affect cell proliferation and found that either ATG4A overexpression or ATG4A knockdown had no effect on the proliferation of gastric cancer cells (Supplementary Figure S3A and B). Collectively, these results indicate that ATG4A promotes the migration and invasion of gastric cancer cells *in vitro*.

**Figure 2:** ATG4A promotes gastric cells migration and invasion *in vitro* **A.** Expression of ATG4A protein in gastric cancer cells (MKN-47, SGC-7901, MGC-823, MGC-803 and MKN-45 cell). The right bar graph represents relative intensity. **B.** Wound healing assay for ATG4A-overexpressed SGC-7901 (ATG4A-OE) cells compared with control cells (NC). The right graph presents the ratios of migrated ATG4A-OE cells relative to those of the control group. **C.** Matrigel™ invasion assay for ATG4A-OE cells compared with NC. The invasion index was calculated between NC cells and ATG4A-OE cells in the right bar graph. **D.** Wound healing assay for ATG4A-knockdown MGC-803 cells (ShATG4A-1, ShATG4A-2, ShATG4A-3) and control cells (Mock). **E.** Matrigel™ invasion assay for knockdown MGC-803 cells and control cells. * *P* < 0.05.

### ATG4A promotes tumor metastasis *in vivo*

A tail vein metastatic assay was performed in nude mice to examine the metastatic potential of ATG4A-OE and ShATG4A-1 cells compared with control cells. As shown in Figure 3, the number of lung metastatic lesions derived from ATG4A-OE cells was markedly increased compared with control cells. The average number and volume of metastatic tumors in the animal lungs following injection with ATG4A-OE cells was high compared to control cells (Figure 3A and 3C). By contrast, ATG4A knock down significantly inhibited the metastatic potential. Mice injected with ShATG4A-1 cells developed fewer and smaller lung metastasis lesions than mice injected with control cells (Figure 3B and 3D). Collectively, these results show that ATG4A could promote tumor metastasis *in vivo*.

The article "ATG4A promotes tumor metastasis by inducing the epithelial-mesenchymal transition and stem-like properties in gastric cells" was retracted in 2025. Reasons: contaminated cell lines or tissues; duplicated images; unreliable data; unreliable results or conclusions.

**Figure 3:** ATG4A promotes the lung metastasis of gastric cancer cells **A.** Representative photographs of lung colonization derived from ATG4A-OE xenograft-bearing mice and control cell (NC) xenograft-bearing mice (Upper panel). The middle and lower panels show representative images of HE and ATG4A IHC staining, respectively. **B.** Representative photographs of lung colonization derived from ATG4A-shRNA (ShATG4A-1) xenograft-bearing mice and control cell (Mock) xenograft-bearing mice (Upper panel). The middle and lower panels show representative images of HE and ATG4A IHC staining, respectively. Red arrows indicate metastatic tumor colonization. **C.** Quantified analysis of the average number and volume of metastatic tumor nodules derived from ATG4A-OE cells and control cells. **D.** Quantified analysis of the average number and volume of metastatic tumor nodules derived from ATG4A-shRNA cells and control cells.

### ATG4A induces the EMT phenotype and stem cell-like properties in gastric cancer cells

Recently, both epithelial-mesenchymal transition (EMT)-type cells and cancer stem cells (CSCs) were believed to be involved in tumor metastasis [19, 20]. Thus, we investigated whether ATG4A regulates EMT and stem cell properties in gastric cancer cells. Reduced E-cadherin (epithelial phenotype) expression and increased vimentin and N-cadherin (mesenchymal phenotype) levels were detected in ATG4A-overexpressing cells, indicating that the stable overexpression of ATG4A induces EMT in SGC-7901 cells (Figure 4A). By contrast, ATG4A knockdown using three individual shRNAs reverted a mesenchymal phenotype to an epithelial phenotype in MGC-803-ATG4A shRNA cells, accompanied with increased E-cadherin expression as well as decreased N-cadherin and vimentin levels (Figure 4B). These data suggest that ATG4A expression may regulate the plasticity between EMT and MET.

To investigate whether ATG4A induces stem cell properties, stem cell markers such as Sox-2, Oct-4 and Bmi-1 were detected [21]. As expected, enhanced ATG4A expression led to significant elevation in the Sox-2, Oct-4 and Bmi-1 levels, while ATG4A knockdown reduced the expression of Sox-2, Oct-4 and Bmi-1, compared with control cells (Figure 4C and 4D). The effect of ATG4A on the sphere formation of gastric cancer cells was also evaluated. As shown in Figure 4, the number and size of spheres formed by ATG4A-overexpressing SGC-7901 cells were increased compared to control cells (Figure 4E). By contrast, ATG4A knockdown reduced the number and size of tumorspheres in MGC-803 cells (Figure 4F). *In vivo*, tumor-initiating capacity of SGC-7901 was increased by ATG4A-overexpression. Similarly, ATG4A knockdown reduced the tumor-initiating capacity of MGC-803 (Figure 4G). These results indicate that ATG4A induces stem cell-like properties of gastric cancer cells.

The article "ATG4A promotes tumor metastasis by inducing the epithelial-mesenchymal transition and stem-like properties in gastric cells" was retracted in 2025. Reasons: contaminated cell lines or tissues; duplicated images; unreliable data; unreliable results or conclusions.

**Figure 4:** ATG4A induces the EMT phenotype and stem cell properties in gastric cancer cells **A.** Protein levels of EMT markers in ATG4A-OE cells and control cells. **B.** Protein levels of EMT markers in ATG4A-shRNA cells and control cells. **C.** Protein levels of stemness markers in ATG4A-OE cells and control cells. **D.** Protein levels of stemness markers in ShATG4A cells and control cells. **E.** Representative images and quantitative analysis show that ATG4A-OE cells formed more tumorspheres. **F.** Representative images and quantitative analysis show that ShATG4A cells formed fewer tumorspheres. **G.** Effect of ATG4A on the tumor initiation capacity of gastric cancer cells. The number of spheres was counted for 6 fields in each group. The data are expressed as the means ±SD, *P < 0.05.

### ATG4A regulates EMT and stemness *via* the Notch pathway, not *via* autophagy

ATG4A plays an important role in the formation of autophagosomes in cells [22, 23]. Thus, we investigated whether autophagy was the underlying mechanism of ATG4A-mediated invasion and metastasis of gastric cancer cells. Interestingly, we observed no change in LC3-I/LC3-II and autophagosome formation after either ATG4A upregulation or ATG4A silencing (Figure 5A and Supplementary Figure S4). There results suggested that ATG4A promotes invasion and metastasis in gastric cancers by an autophagy-independent mechanism.

The maintenance of CSCs and EMT phenotypic cells is regulated by signaling pathways, including the Notch, Hedgehog, Wnt, PDGF, Akt, TGF-β, NF-κB and miRNA [20]. To further explore which pathway participated in ATG4A-induced EMT and promoted stemness in gastric cancer cells, several key molecules involved in signaling pathways, such as the Notch signaling, Wnt signaling, TGF-beta signaling and NF-κB signaling pathways, were detected. As shown in Figure 5B and 5C, ATG4A inhibition resulted in the decreased expression of the Notch signaling pathway-targeting molecule Hes-1, while ATG4A overexpression upregulated Hes-1 expression. These results showed that ATG4A induced EMT and stemness by activating the Notch signaling pathway. To further investigate whether the Notch pathway was necessary for ATG4A-induced EMT and stemness, DAPT, the Notch signaling inhibitor, was used to treat ATG4A-OE gastric cancer cells, and both EMT and stemness markers were analyzed. As shown in Figure 5D, DAPT treatment significantly decreased the levels of vimentin, Sox-2 and Hes-1, but upregulated the levels of E-cadherin, in ATG4A-OE cells. In addition, DAPT significantly inhibit the migration and invasion capacity of ATG4A overexpression gastric cancer cells (Figure 5E and 5F). Taken together, these results indicate that ATG4A regulates both EMT and the stemness of gastric cancer cells through the Notch signaling pathway, not through autophagy.

The article "ATG4A promotes tumor metastasis by inducing the epithelial-mesenchymal transition and stem-like properties in gastric cells" was retracted in 2025. Reasons: contaminated cell lines or tissues; duplicated images; unreliable data; unreliable results or conclusions.

**Figure 5:** Notch signaling is involved in the ATG4A-induced EMT and stemness of gastric cancer cells **A.** Knockdown or upregulation of ATG4A has no effect on the autophagic flux in gastric cancer cells. The protein levels of LC3-I, LC3-II and ATG4A were determined by Western blotting. The right panel is the quantitative data of ATG4A and LC3-II/LC3-I, with β-actin as the normalization control. **B.** Quantitative PCR analysis of Wnt-5a, Hes-1, NF-KB and Smad-3 gene expression in ATG4A overexpression or knockdown gastric cancer cells. **C.** Western blot of HES-1 in ATG4A overexpression or knockdown gastric cancer cells. **D.** Western blot analysis of ATG4A, Hes-1 (Notch downstream gene), E-cad (EMT marker), Vim and Sox2 (stemness marker) in ATG4A-overexpression gastric cancer cells in the presence or absence of the γ-secretase inhibitor (DATP). **E.** The scratch assay was used to detect the effect of DNTP on the migration ability of gastric cancer cells overexpressing ATG4A. **F.** The transwell assay was used to detect the effect of DATP on the invasion ability of gastric cancer cells overexpressing ATG4A. The data are expressed as the means ±SD, *P < 0.05.

## DISCUSSION

Cancer cells with stem-like properties are proposed to play important roles in tumor metastasis by acquiring the epithelial-mesenchymal transition (EMT) phenotype. Thus, targeting EMT pathways and CSC maintenance are believed to be promising therapeutic strategies. In this study, we first demonstrated that both gastric cancer cells in the invasive frontier area and metastatic lymph nodes expressed high levels of ATG4A compared with primary cancer cells. ATG4A overexpression induced EMT and stem cell properties both *in vitro* and *in vivo* through activation of the Notch pathway but not *via* autophagy. These results indicate that ATG4A is a potential target for gastric cancer treatment.

The article "ATG4A promotes tumor metastasis by inducing the epithelial-mesenchymal transition and stem-like properties in gastric cells" was retracted in 2025. Reasons: contaminated cell lines or tissues; duplicated images; unreliable data; unreliable results or conclusions.

ATG4 protein belongs to the cysteine protease family, which, in conjunction with phosphatidylethanolamine, can lead to the recycling of ATG8. This recycling is required for the formation of double-membrane autophagosomes [22, 24, 25]. Four subtypes of ATG4 proteins have been reported in yeast *Saccharomyces cerevisiae*, and two homologs, ATG4A and ATG4B, have been found in the human genome [22, 26]. ATG4B-knockout mice display reduced autophagic activity [27]. More recent studies have reported that ATG4B serves as an oncogene to promote tumorigenesis in colorectal cancer cells [28]. However, little is known about the physiological function of ATG4A in autophagy and tumorigenesis. Recent studies have shown that ATG4A participates in VP16-DDP resistance in small cell lung cancer through Mir-24-3p, and the reduction of ATG4A protein expression by the overexpression of Mir-24-3p allows small cell lung cancer cells to be resensitized to VP16-DDP [17]. In this study, we found that the ATG4A protein is upregulated in gastric cancers, especially cells in the invasive frontier area and lymph node metastatic lesions compared with matched normal tissues. Moreover, ATG4A expression was positively related with the previously reported lymph node metastasis biomarkers VEGF-C, suggesting ATG4A play an important role in regulating gastric cancer metastasis (Figure S5). Cancer cells escape the primary tumor mass and colonize new areas in the body by a series of processes, including migration, invasion, entrance into the circulatory system, travel to a distant site, proliferation and formation of new colonies [29]. Lymph node metastasis is an initial step of gastric cancer metastasis, and lymph node metastasis is considered an important prognostic factor in gastric cancer patients [30–32]. Our results that lymph node metastatic lesions express higher levels of ATG4A suggest that ATG4A is involved in the development and acquisition of a migratory and invasive cell phenotype in gastric cancer cells. The role of ATG4A in migration, invasion and metastasis was further validated *in vitro* and *in vivo*. Our results suggest that ATG4A is a promoter of gastric cancer development and metastasis.

EMT is a key program during morphogenesis and cancer progression [33], and a fundamental process for cancer cells to leave the primary carcinoma by promoting invasion and metastasis [34]. In this study, we found that ATG4A promoted gastric cancer cell migration by inducing EMT. However, the growth of micro-metastases into macroscopic metastases relies on the properties of self-renewing stem cells. The cells leaving a primary tumor and disseminating into distant sites must have self-renewal capability and proliferative potential [35]. A recent study also revealed a direct link between EMT and stem cell properties [19]. CD44 has been used as an important cell surface markers to sort GCSCs [36]. However, Rocco A et al. found that CD44 do not identify cancer stem cells in primary human gastric tumors [37]. Thus, we selected Sox-2, Oct-4 and Bmi-1 as gastric cancer stem markers [38]. Our study demonstrates that ATG4A overexpression induces the expression of Sox-2, Oct-4 and Bmi-1 in gastric cancer cells. By contrast, ATG4A knockdown decreased the expression of gastric cancer stem markers. In addition, ATG4A promoted the formation of tumorsperes *in vitro* and tumor-initiating capacity *in vivo*. Taken together, our study indicated that ATG4A can induce the EMT and stemness of gastric cancer cells.

The article "ATG4A promotes tumor metastasis by inducing the epithelial-mesenchymal transition and stem-like properties in gastric cells" was retracted in 2025. Reasons: contaminated cell lines or tissues; duplicated images; unreliable data; unreliable results or conclusions.

The molecular mechanism of ATG4A regulation EMT and stemness was further explored. Increased ATG4A expression is required for autophagosome fusion in early differentiating human erythroblasts [15]. ATG4A can cleave MAP1LC3, GABARAP, GABARAPL2 and ATG8 *in vitro*, which are required for autophagosome biogenesis phagophore elongation and autophagosome sealing, respectively [28, 39]. In our study, we detected no changes in LC3-II or LC3-I expression and autophagosome formation after either upregulation or silencing of ATG4A expression *in vitro*, suggesting that ATG4A induced the EMT and stemness of gastric cancer cells in an autophagy-independent manner. This result may be explained by a previous study that ATG4B plays more important roles in the autophagic process than ATG4A [40].

The Notch signaling pathway is involved in cell proliferation, survival, apoptosis, and differentiation and plays an important role in the development and progression of several malignancies [41–43]. A recent study found that the Notch signaling pathway also regulates EMT and tumor aggressiveness [44]. Notch-1 induces the EMT phenotype of cancer cells by repressing E-cadherin expression and upregulating Snail and Slug expression [45–47]. EMT has been mechanistically linked to stem-like signatures regulated by Notch-1 in prostate cancer cells [48]. In colorectal cancer patient specimens, Notch-1 was found to be up-regulated in colon tumor tissue and to increase the abundance of EMT- and stemness-associated proteins, such as CD44, Slug and Smad-3 [49]. These studies indicated that the Notch pathway was associated with the EMT and acquisition of stem cell-like properties in cancer cells. In this study, we found that Hes-1, a key downstream molecule of Notch signaling, was exclusively upregulated by ATG4A overexpression. Furthermore, the increased expression of EMT and stemness markers induced by ATG4A overexpression was reversed by the Notch signaling inhibitor DAPT. These results indicate that the EMT phenotype and stemness properties induced by ATG4A depend on activation of the Notch signaling pathway. During the activation of Notch receptors, they are cleaved by metalloprotease and γ-secretase, generating extracellular (NECD) and intracellular (NICD) fragments [50]. Next, the NICD translocates to the nucleus, leading to the activation of Notch-associated gene expression [51]. ATG4A is a cysteine protease. Whether ATG4A could activate Notch signaling by releasing NICD from the transmembrane needs to be further investigated.

The article "ATG4A promotes tumor metastasis by inducing the epithelial-mesenchymal transition and stem-like properties in gastric cells" was retracted in 2025. Reasons: contaminated cell lines or tissues; duplicated images; unreliable data; unreliable results or conclusions.

Taken together, we demonstrate that ATG4A promotes tumor metastasis by inducing EMT and the stem-like properties of cancer cells through the activation of Notch signaling, not through autophagy. Our findings suggest that ATG4A is a novel indicator of invasion and metastasis in gastric cancer and can be a potential candidate target for the treatment of gastric cancer.

## MATERIALS AND METHODS

### Gastric cancer specimens and patient characteristics

Surgical specimens involved in the study were obtained from 110 patients (67 men and 43 women) with histologically confirmed gastric cancer who accepted curative resection during 2010 at Southwest Hospital (Third Military Medical University, Chongqing). Those patients who received neo-adjuvant therapy prior to surgery were not included. Formalin-fixed paraffin-embedded tissues were used for immunohistochemical staining. The tumor stage was determined according to the TNM classification system of the International Union against Cancer (UICC) [52]. Histological differentiation was determined according to the criteria of the World Health Organization. In our research, we chose the tumor tissues, lymph node, and junctional zone. Adjacent tissue that was free from cancer cells was used as a control. All 110 patients or their guardians provided written informed consent to use excess pathological specimens for research. This study was conducted according to the principles of the Helsinki Declaration and was approved by the ethics committees of the Third Military Medical University (TMMU).

### Immunohistochemistry and evaluation of immunohistochemical staining

Paraffin-embedded tissues were sliced into 4-μm-thick sections. The sections were then deparaffinized, rehydrated, and blocked by peroxidase with 3% H_2_O_2_ in methanol for 30 min at 37°C. Antigen retrieval was performed by transferring the sections into Tris-acetate-ethylenediamine tetraacetic acid (EDTA) buffer (pH 8.0) inside a 700-watt microwave oven on full power for 5 min and half power for 15 min. After cooling to room temperature, the sections were blocked in goat serum for 1 h and were incubated with anti-ATG4A (1:400; Rabbit monoclonal, Abcam, USA) antibody at 4°C overnight. Next, the sections were incubated with biotinylated secondary antibody (1:2000) for 1 h at 37°C, followed by washing in PBS and then visualization using the DAB Color Developing Reagent Kit. Negative control group and positive control group were used to test the antibody specificity [16]. The tissues were observed under the Olympus BX51 microscope. The ATG4A level was evaluated by scores defining staining areas and intensity. The staining area was scored as follows: 0 = no ATG4A-positive cells; 1 = < 25% positive cells; 2 = 25% to 50% positive cells; and 3 = 50% to 75% positive cells; 4 = >75% positive cells. The staining intensity was scored as 1, 2 and 3 according to the intensity of the positive ATG4A reaction: a score of 1 was defined as low expression, a score of 2 was defined as moderate expression, and a score of 3 was defined as high expression. The total score was calculated by the formula: Score = area score × intensity score. The scoring of the specimens was performed by two independent pathologists.

The article "ATG4A promotes tumor metastasis by inducing the epithelial-mesenchymal transition and stem-like properties in gastric cells" was retracted in 2025. Reasons: contaminated cell lines or tissues; duplicated images; unreliable data; unreliable results or conclusions.

### Cell culture

The human gastric cancer cell lines MKN-47, SGC-7901, MGC-823, MGC-803, and MKN-45 were used in this study. All of the cell lines were obtained from American Type Culture Collection and were cultured in DMEM medium (Gibco/Invitrogen, Grand island, NY) containing 10% fetal bovine serum (HyClone, Logan, UT) in 5% CO_2_ at 37°C. The images of gastric cancer cell lines were acquired by an Olympus inverted microscope.

### Overexpression and knockdown of ATG4A using lentivirus

Lentiviral constructs expressing or repressing ATG4A were cloned into the Plvx and PLKO.1 vector backbone. Cloning and virus production were performed following the protocol provided by the manufacturer (Cellecta, Mountain View, CA). Viral supernatant was harvested for 48 h post transfection and separated from debris *via* centrifugation. For ATG4A overexpression, the lentiviral-ATG4A and control lentivirus were infected into SGC-7901 cells for 24 h in medium containing 6 μg/ml polybrene (Sigma-Aldrich, St. Louis, MO). For ATG4A knockdown, the three ATG4A shRNA lentivirus and control lentivirus constructs were infected into MGC-803 cells, and stable transfectants were selected with 2.5 μg/ml puromycin (Sigma-Aldrich) for 48 h. Following selection, the cells were recovered for 48 h in antibiotic-free culture medium to establish cells stably expressing or repressing ATG4A.

The article "ATG4A promotes tumor metastasis by inducing the epithelial-mesenchymal transition and stem-like properties in gastric cells" was retracted in 2025. Reasons: contaminated cell lines or tissues; duplicated images; unreliable data; unreliable results or conclusions.

### Cell proliferation assay

Cell proliferation analysis was performed on SGC-7901 and MGC-803 cells, which were expressing ATG4A siRNA, over-expression, or negative control constructs. These cells were cultured in 96-well microtiter plates and the cell proliferation rates analyzed using a MTT Cell Proliferation Assay Kit (Thermo Scientific, USA). All of the results were derived from 6 sets of duplicated experiments.

### Cell migration and invasion assays

Cell migration assays were performed with Transwell chambers (8-μm pore size) (Corning, Acton, MA) according to the manufacturer's instructions. Cells (5 × 10^4^) were placed onto the top chamber of each insert for the tumor cell invasion assay. Similar inserts coated with a mixture of Matrigel™ (BD Biosciences, San Jose, CA) and DMEM (1:1, v/v) were used to determine the invasive potential for tumor cell invasion assays. After incubation for 36 h at 37°C, the Transwell chambers were removed from the plates and fixed with 4% paraformaldehyde. Non-migrating or noninvasive cells on the upper surface of the Transwell chambers were then removed with a cotton swab, and the remaining cells were stained with crystal violet solution. Cell numbers were counted in five randomly fields in each Transwell chamber under a light microscope at ×200 magnification.

### Wound healing assay

Cells were seeded in six-well plates to measure two-dimensional movement. A wound was created with a sterile pipette tip in the middle of a confluent plate. Next, the medium was replaced with DMEM medium without FBS. Photographs were captured immediately or after 36 hours using an Olympus BX51 microscope, and the wound distance was calculated as a basic width. Wound closure (%) was determined as the width migrated after 36 hours relative to the basic width.

### Tumorsphere formation assay

For the self-renewal assay, cells were cultured and suspended in serum-free DMEM/F12 medium (Gibco/Invitrogen) supplemented with 20 ng/mL basic fibroblast growth factor (FGF) (Sigma-Aldrich), 20 ng/mL EGF (Sigma-Aldrich), and 1× B27 (Invitrogen, Carlsbad, CA). The cells were seeded in 24-well ultra-low attachment plates (Corning) to acquire tumorspheres. The number of primary gastric cancer cell spheres was counted after 2 weeks under a microscope at ×200 magnification in 5 random fields, and pictures were taken. Each experiment was performed in triplicate.

### Quantitative real-time PCR

Total RNAs were extracted using Trizol™ reagent (Invitrogen, USA). First-strand cDNA was synthesized for each sample using the PrimeScript RT Reagent Kit (Perfect Real Time) (Takara Bio Inc., Kusatsu, Shiga, Japan). For the detection of the expression levels of Wnt-5a, Hes-1, NF-κB, Smad-3 and GAPDH, PCR was performed using the CFX96 Real-Time PCR system (Bio-Rad Laboratories, Hercules, CA) and SYBR Premix Ex Taq II (Bio-Rad). The primers used in our study are listed in Supplementary Table S1. The relative gene expression levels were calculated using the 2-comparative Ct ^(2-ΔΔCt)^ method, and the mRNA expression levels were normalized against the threshold cycle (C_t_) of GAPDH.

The article "ATG4A promotes tumor metastasis by inducing the epithelial-mesenchymal transition and stem-like properties in gastric cells" was retracted in 2025. Reasons: contaminated cell lines or tissues; duplicated images; unreliable data; unreliable results or conclusions.

### Western blot analysis

Total proteins were extracted using RIPA lysis buffer on ice, electrophoresed on 12% SDS-PAGE gels (Bio-Rad) and blotted onto nitrocellulose membranes (Amersham Biosciences Corp, Sunnyvale, CA). The membranes were blocked with 5% non-fat milk powder at room temperature for 2 hours and incubated overnight with primary antibodies: anti-ATG4A (1:400) (Abcam, Cambridge, UK), anti-E-cadherin (1:2000) (BD Transduction Laboratories, Franklin Lakes, NJ), anti-N-cadherin (1:1000) (BD Transduction Laboratories), anti-vimentin (1:1000) (BD Transduction Laboratories), anti-Sox2 (1:500) (Abcam), anti-Oct4 (1:400) (Abcam), anti-Bmi-1 (1:400) (Abcam), anti-LC3I/II (1:1000) (Cell Signaling Technology, Danvers, MA) and anti-β-actin antibody (1: 2000) (Sigma-Aldrich). After three 5-min washes, the membranes were incubated with horseradish peroxidase (HRP)-conjugated secondary antibodies (1: 2000) (Santa Cruz Biotechnology, Dallas, TX) for 2 hours at room temperature and then washed again in TBS-T and visualized with an enhanced chemiluminescence kit (ECL-kit) (Santa Cruz Biotechnology). All of the experiments were performed in triplicate.

### Transmission electron microscopy

Standard transmission electron microscopy (TEM) was applied for ultrastructural analysis. The cells were fixed and embedded. Thin sections (90 nm) were cut and examined at 80 kV using a JEOL 1200EX transmission electron microscope. Approximately 5 cells were counted, and autophagosomes were defined as structures measuring 2.0 μm.

### Animal experiments

For *in vivo* metastasis assays, 2×10^6^ cells stably transfected with overexpressing ATG4A, Sh-ATG4A or control cells were injected into nude mice (five per group, 4- to 6-week-old male BALB/c-nu/nu) through the tail vein. The mice were sacrificed after 7 weeks, and lung tissues were dissected and fixed by phosphate-buffered neutral formalin paraffin embedding. The paraffin blocks were detected by hematoxylin and eosin staining and immunohistological staining with ATG4A. Metastatic tumors were quantified by counting metastatic lesions in each section. And the average volume of tumor was quantified by the maximum diameter of tumor. Cells at limiting dilution (1 ×105, 1 × 104 and 1 × 103) were injected into BALB/c nude mice within Matrigel, the tumour initiation was calculated. All of the animal experiments were approved by the Institutional Animal Care and Use Committee of the Southwest Hospital, TMMU, according to the Guide for the Care and Use of Laboratory Animals.

The article "ATG4A promotes tumor metastasis by inducing the epithelial-mesenchymal transition and stem-like properties in gastric cells" was retracted in 2025. Reasons: contaminated cell lines or tissues; duplicated images; unreliable data; unreliable results or conclusions.

### Statistical analysis

All of the statistical analyses were performed using the SPSS 18.0 statistical software program. The quantitative values of all experiments were presented as the mean ± SD and were calculated from 3 independent experiments. The data were analyzed by Student's t test. For immunohistochemistry assays, the difference in the expression level of ATG4A was calculated according to the IRS score, and the relationships between ATG4A expression and clinicopathologic characteristics were performed using Fisher's exact test. A P value less than 0.05 was considered to be statistically significant.

## SUPPLEMENTARY MATERIAL FIGURES AND TABLE


